# Robot-Assisted Gait Training Plan for Patients in Poststroke Recovery Period: A Single Blind Randomized Controlled Trial

**DOI:** 10.1155/2021/5820304

**Published:** 2021-08-29

**Authors:** Deng Yu, Zhang Yang, Liu Lei, Ni Chaoming, Wu Ming

**Affiliations:** The First Affiliated Hospital of USTC, Division of Life Sciences and Medicine, University of Science and Technology of China, Hefei, Anhui 230001, China

## Abstract

**Background:**

Walking dysfunction exists in most patients after stroke. Evidence regarding gait training in two weeks is scarce in resource-limited settings; this study was conducted to investigate the effects of a short-term robot-assisted gait training plan for patients with stroke.

**Methods:**

85 patients were randomly assigned to one of two treatment groups, with 31 patients in withdrawal before treatment. The training program comprised 14 2-hour sessions, for 2 consecutive weeks. Patients allocated to the robot-assisted gait training group were treated using the Gait Training and Evaluation System A3 from NX (RT group, *n* = 27). Another group of patients was allocated to the conventional overground gait training group (PT group, *n* = 27). Outcome measurements were assessed using time-space parameter gait analysis, Fugl-Meyer Assessment (FMA), and Timed Up and Go test (TUG) scores.

**Results:**

In the time-space parameter analysis of gait, the two groups exhibited no significant changes in time parameters, but the RT group exhibited a significant effect on changes in space parameters (stride length, walk velocity, and toe out angle, *P* < 0.05). After training, FMA scores (20.22 ± 2.68) of the PT group and FMA scores (25.89 ± 4.6) of the RT group were significant. In the Timed Up and Go test, FMA scores of the PT group (22.43 ± 3.95) were significant, whereas those in the RT group (21.31 ± 4.92) were not. The comparison between groups revealed no significant differences.

**Conclusion:**

Both the RT group and the PT group can partially improve the walking ability of stroke patients within 2 weeks.

## 1. Introduction

Stroke is a major cause of disability. Previous studies have reported that, 3 months after onset, one-third of surviving patients remain wheelchair-dependent and gait velocity and endurance are significantly reduced in approximately 80% of ambulatory patients [1–3]. Therefore, to aid patients' subsequent return to society, restoring walking function is the main goal of early rehabilitation [4].

To date, the most effective treatment options (frequency and duration) for improving gait early after stroke, as well as apparent improvement and duration, are still the subject of debate [5]. On the one hand, it has been observed that repetitive task-specific methods with higher walking intensity can lead to greater improvement in the gait of stroke patients [6]. Specifically, it was reported that people who received a combination of electric-assisted gait training and physical therapy after a stroke exhibited greater improvement than those who received only regular gait training, especially in the first 3 months after stroke, and were more likely to achieve independent walking [7]. On the other hand, for subacute stroke participants with moderate to severe gait disorder, the variety of conventional gait training interventions is reported to be more effective than robot-assisted gait training [8, 9]. In addition, there is evidence that gait performance will be improved regardless of whether walking training uses robotic gait training or ground exercise [10].

Since the end of 2019, according to China's domestic and local medical insurance policies, in most parts of China, if medical insurance is used to repay hospitalization expenses, stroke patients can only be hospitalized for 2 weeks. Because the conventional 4-week hospital stay has been reduced to 2 weeks, it is important to develop more accurate and effective rehabilitation methods for early stroke patients. To examine this issue, we compared the effects of an early treatment plan involving robotic gait training (RT) with conventional overground gait training (PT) to determine the most beneficial treatment plan for gait improvement.

## 2. Methods

### 2.1. Study Design

This was a single-center, single blind, randomized controlled trial. The study was approved by the First Affiliated Hospital of University of Science and Technology of China (IRB, Institutional Review Board) (No. 2020-KY627). The inclusion criteria were as follows: first middle cerebral artery stroke (documented by a computerized tomography scan or magnetic resonance imaging); time from stroke onset of less than 12 weeks; Brunnstrom stage of lower extremity function which was from stage III to stage IV; Montreal Cognitive Assessment (MoCA) score ≥ 26 points, able to cooperate with completion of rehabilitation training and able to clearly express feelings about the training [11]; aged 35-75 years, male or female; and agreement to participate in the clinical trial, providing written informed consent.

The exclusion criteria were as follows: transient ischemic attack; previous brain lesions, irrespective of etiology; presence of neglect evaluated using the Bells Test (a difference of five of 35 bells omitted between the right and the left sides indicates hemispatial neglect) [12, 13]; aphasia; neurological examination to assess the presence of clinically relevant somatosensory impairment; severe spasticity affecting the lower extremities (modified Ashworth scale score greater than 2); clinical examination to assess the presence of lower extremity motor apraxia (with movement errors of limb movement types classified using the following criteria: awkward movements in the absence of basic movements and sensory deficits, ataxia, and normal muscle tone); involuntary automatic dissociation; lower limb skeletal variations, deformities, anatomical abnormalities, and joint impairment with various causes; local skin infection or damage below the hip joint of the lower limb; patients with epilepsy, in which their condition had not been effectively controlled; combination of other serious systemic diseases, such as severe cardiopulmonary dysfunction; participation in other clinical trials within 1 month before the trial; and failure to sign informed consent. All subjects were volunteers, and all provided written informed consent to participate in the study, which was carried out according to the Declaration of Helsinki and approved by the Ethics Committee of the First Hospital Affiliated to the University of Science and Technology of China.

Before the test, we randomly assigned eligible participants to two groups. We assigned patients to one of two treatment groups based on the restricted randomization scheme generated by the software. Investigators who determined whether a patient was eligible for inclusion in the trial did not know which group (hidden assignment) the patient would be assigned to when making their decision. Another investigator checked the correct allocation of patients according to the randomization table. Besides the treatments included in the study protocol, the two groups of patients received 0.5 hours of conventional physiotherapy every day, and no other type of rehabilitation was performed.

#### 2.1.1. RT Group

Patients assigned to this group underwent gait training through the Gait Training and Evaluation System A3 (NX, China), which is a driven electromechanical gait robot that provides repeatable, high-intensity, and task-specific gait training. Automated exercise training was conducted on treadmills. Patients who did not participate in the assessment underwent supervised treatment with adjusted treadmill speed and weight support. This system involved dynamic and static weight loss systems, which can simulate real center of gravity changes when walking. As functions improve, the levels of weight support, treadmill speed, and guidance force are all adjusted to maintain the weak side of the knee extensor muscles during the standing position. The weight support level is gradually reduced from 50% to 0%, and the guiding force is reduced from 100% to 10% (by reducing the guiding force, which is used in both the standing and swinging phases, the patient is forced to use the hip and knee muscles to participate more actively in the gait process) [14, 15]. In addition, according to the tolerance of each patient, the treadmill speed (from 1.2 km/h) increased by 0.2 to 0.4 km/h per course of treatment, up to 2.6 km/h. The effective duration for each RT was 50 minutes.

#### 2.1.2. PT Group

Conventional overground gait training is based on traditional neurodevelopmental therapy techniques. This therapy involved practicing sitting-standing balance, active transfer, sitting-standing, and intensive training for patients with sensorimotor disorders. With the improvement of physical functioning, the training of patients further increased in difficulty, including dynamic standing balance training, finally developing into functional gait training, while continuing to carry out intensive training [16].

Patients were assigned to this group for ground gait training (effective time of 50 minutes per lesson), aimed at improving posture control during gait, weight transfer, standing phase, free swing phase stability, heel full contact, and gait mode. The same trained therapist treated all patients in this group and standardized the performance of each exercise according to the patient's skills (i.e., ability to participate in a progressive and more active manner during gait) and tolerance intensity, as previously described for the RT group.

### 2.2. Procedures

All participants underwent a training program consisting of a 2-hour course (including rest period) each day for 14 consecutive days. Each training session consisted of two 50-minute training periods, with one 20-minute rest period between them. Patients were evaluated at baseline and after 1 week and 2 weeks (primary endpoint). The same rater did not have knowledge of the group assignment and evaluated all patients. We tested the effectiveness of the blinding procedure by asking the evaluator to make an educated guess.

### 2.3. Outcomes

The main results were FMA scores and TUG test scores before and after training. Time-space parameter gait analysis was also conducted using a balance function assessment system (model: AL-080, Anhui Aili Intelligent Technology Co, Anhui, China) [17], including stride time (s), single stance phase time (s), double stance phase time (s), swing phase time (s), stance phase time (s), stride length (cm), walk velocity (m/s), cadence (steps/min), gait width (cm), and toe out angle (deg).

In this study, the symmetry ratio between the bilateral space/time parameters can be used to easily identify the degree of symmetry between the affected side and the less affected side. The formula for the symmetry ratio obtained from the symmetry ratio is as follows [18]:

(1) $$\begin{array}{c} \text{Symmetry ratio}=\frac{\text{affected side }\left(\text{parameter value}\right)}{\text{less affected side }\left(\text{parameter value}\right)}. \end{array}$$

When the affected side is symmetrical to the less affected side, the result of the symmetry ratio is 1. When the symmetry ratio is greater than 1, the parameter distribution corresponding to the affected side is relatively high. When the symmetry ratio is less than 1, the parameter distribution corresponding to the less affected side is higher.

### 2.4. Statistical Analysis

SPSS statistical analysis software 18.0 was used to analyze the data. The Kolmogorov-Smirnov test was used to assess the assumption of normality. The characteristics of the participants in each group were tested using independent *t*-tests for normally distributed variables and Mann–Whitney *U* tests for nonnormally distributed variables. The Wilcoxon signed rank test was used to compare the changes before and after treatment between the two groups. *P* values < 0.05 were considered to indicate statistical significance.

## 3. Results

From April 2020 to December 2020, a total of 85 volunteers who met the eligibility criteria with chronic stroke signed up to participate in the experiment. They were randomly assigned to the PT group (*n* = 40) and the RT group (*n* = 45). 31 patients did not receive the assigned intervention (withdrawal before treatment) and could not be treated for various personal reasons and the limitations of the clinical screening conditions. In the end, 54 participants who met the eligibility criteria participated in the training (PT group, *n* = 27; RT group, *n* = 27). A mixed flow chart depicting the research design is shown in Figure 1. No serious adverse events or major hazards were reported.

### 3.1. Baseline

At the baseline assessment, no significant differences were observed between the two groups in terms of age (*P* = 0.14), stroke onset time (*P* = 0.47), FMA scores (*P* = 0.06), and TUG scores (*P* = 0.17). The demographic and clinical characteristics of patients are shown in Tables 1 and 2.

### 3.2. Outcome

Thus, the final analyses included 54 patients: 27 in the RT group and 27 in the PT group. Age, weeks poststroke, sex, side of stroke, and stroke type did not differ significantly between the two groups (see Table 1). We measured improvement by calculating the difference between the baseline and 2-week scores of each group. Because the data were not normally distributed, the Mann–Whitney *U* test was used to compare baseline and posttraining measurements between the two groups. There were no significant differences between groups in any outcome measurements before treatment.

After 14 training sessions, both groups showed significant improvements in at least one outcome measure. Moreover, the PT group exhibited a significantly greater performance improvement (see Table 2). Regarding FMA and TUG scores, the comparison of scores before and after 2 weeks of training revealed significant differences within the PT group (*P* < 0.01) (see Table 2) and significant differences in the RT group (FMA, *P* = 0.02), but the results of TUG (*P* = 0.28) exhibited no difference. The comparison between groups showed that there was no significant difference between the two groups in FMA scores (*P* = 0.26) or TUG scores (*P* = 0.97).

Regarding the time parameter gait analysis, in the intragroup comparison, there were no significant differences before and after each part of the two groups affected side (*P* > 0.05). In the intragroup comparison of the contralateral swing phase, the RT group was statistically significant (*P* = 0.01). In the symmetry of both sides of the lower limbs before and after two weeks of training in the standing period and swing period, the RT group was statistically significant in the intragroup analysis (*P* = 0.04). In addition, the stance phase, swing phase, and symmetry ratio of the less affected side and the affected side were not significant within and between groups (*P* > 0.05) (see Figure 2).

Regarding the space parameter gait analysis, before and after 2 weeks of training, there was a significant difference in gait width on the affected side (*P* = 0.02) in the PT group. In the RT group, the affected side exhibited significant differences in walking velocity (*P* = 0.03), toe out angle (*P* = 0.01), and stride length (*P* = 0.03). However, after 14 days of training, the two groups did not exhibit any significant improvement in cadence. Except for the significant statistical difference in toe out angle (*P* = 0.002), no significant differences were revealed in the comparison between groups.

## 4. Discussion

The main purpose of this randomized controlled trial was to compare the effects of robot-assisted gait training (RT group) and conventional ground gait training (PT group) for early stroke patients with gait disorder. The current findings revealed that, compared with conventional ground gait training (PT group), gait training with the A3 robot using NX had several key advantages for improving motor function.

Several previous studies have reported that robotic gait training combined with physical therapy after stroke increased the likelihood of achieving independent walking compared with gait training without these devices, and people receiving this intervention in the first 2 months after stroke and those who could not walk were found to benefit the most [19, 20]. Our initial hypothesis was that robot-assisted gait training would be more effective than traditional ground gait training in improving athletic ability, by providing accurate and symmetrical walking patterns to regulate patients' walking. In addition, we predicted that early robot-assisted training after stroke (i.e., dynamic regulation from the weight loss system, real-time adjustment of guidance force, and active and passive training at any time) would be more beneficial than traditional training based on information presented in clear language. Furthermore, we also speculated that gait training with the A3 robot in an upright position would activate the musculoskeletal and cerebrovascular systems through repeated and precise walking posture input, thereby alleviating spastic hypertonia and hyperreflexia and promoting early recovery from stroke.

The current findings did not fully confirm our initial hypotheses. FMA scores revealed that both groups showed significant improvements. In addition, in the early phase, the use of the robotic device to train the spatial parameters of gait led to significantly better performance than traditional ground rehabilitation training. After robot-assisted gait training, patients may not have been able to implement standardized gait quickly and skillfully, and patients' time and space parameters were slightly higher than before training (although this difference was not significant, *P* > 0.05), with no significant difference in TUG scores before and after training (*P* = 0.28). However, regardless of the method, 2 weeks of continuous training did not change the time parameters in patients' gait or step frequency in the space parameters.

The current findings are consistent with some previous reports, supporting the notion that the role of electromechanical/robot equipment is still unclear [10]. Some previous studies' research has suggested that robotic gait training could play an early role in neurorehabilitation, providing correct sensory input as the premise of neural plasticity and the basis of motor learning, which is essential for achieving appropriate motor output [21]. Patients who received a combination of electrically assisted gait training and physical therapy after stroke were more likely to achieve independent walking compared with those who received only conventional gait training, especially in the first 3 months after stroke [7, 14]. In addition, some studies have shown that relying on robot training can improve walking of patients after stroke. In a study by Kim et al., 48 patients within 1 year of illness were divided into a robot-assisted treatment group (0.5 hours of robot training + 1 hour of physical therapy) and a conventional treatment group (1.5 hours of physical therapy), with both groups receiving 1.5 hours of treatment per day. Compared with traditional physical therapy alone, the results revealed that combining robotic devices with physical therapy was superior to conventional therapy in terms of autonomy and balance [22].

However, Mayr and colleagues conducted a study of 66 adult patients with an average of 5 weeks after stroke to evaluate the impact of two groups receiving 8 weeks of inpatient rehabilitation treatment focused on gait ability and gait rehabilitation (robot-assisted gait training and traditional ground gait training). It was reported that, although it took time and energy to achieve beneficial effects of gait training exercise, both methods improved gait function [15]. Similarly, Duncan et al. examined the effects of early exercise training (2 months after stroke onset), late exercise training (6 months after stroke onset), and a home exercise plan (2 months after stroke onset) to study weight-supported running after stroke, including the optimal timing and effectiveness of the mechanical rehabilitation intervention. It was found that, among 408 adult patients with stroke (2 months after stroke), exercise training, including the use of treadmill training for weight support, was no better than exercise therapy performed by a physical therapist at home [8]. Hidler and colleagues proposed a multicenter RCT study that included 72 adult patients less than 6 months after the onset of stroke. The authors report that in individuals with moderate to severe gait disorder after a subacute unilateral stroke, the use of traditional rehabilitation strategies can achieve greater speed and distance on the ground than robot-assisted gait training (using Lokomat devices) [9]. In our study, it can be seen from the comparison between the groups that, except for the significant statistical difference in toe out angle, in fact, the treatment effect of the PT group is similar to that of the RT group in most aspects. Especially in terms of gait width, after 2 weeks of PT training, the intragroup comparison is significant (*P* = 0.02). This reminds us that in rehabilitation training centers without robot training conditions, gait training with conventional overground gait training can also achieve a certain therapeutic effect.

In terms of clinical implications, the current findings tentatively suggest that, for clinical gait training for early stroke, when the patient's gait width is problematic, conventional overground gait training should be chosen; in contrast, when the patient's space parameters (step length, pace, and toe angle) or time parameters (stance phase symmetry ratio) reveal a gait problem, choosing robot-assisted gait training may be more appropriate. However, the main limitation of the current randomized controlled trial was the relatively short training time (2 weeks), limiting the conclusions that can be drawn from our findings. It is possible that training differences between the two methods would be revealed after 4 weeks. A second limitation is related to the study population. The current study was conducted with patients with subacute strokes of different levels of severity, and we were not able to distinguish between spontaneous rehabilitation (means spontaneous recovery of the body) and therapeutic rehabilitation. The selection period (8 weeks) from the onset of stroke was relatively long, possibly involving an excessive number of different spontaneous evolution curves and individual resistance to (training) stress. Another important limitation is the lack of long-term measurement points (e.g., 6 months or more and ideally 1 year). Moreover, starting treatment (i.e., RT) early may not result in a measurable difference in short-term results, even if it does achieve a difference in long-term results.

## 5. Conclusion

This preliminary study shows that both A3 robot-assisted gait training and conventional ground gait training can partially improve the walking ability of stroke patients within 2 weeks.

## Figures and Tables

**Figure 1:** The consort flow diagram of the study.

**Figure 2:** The blank bar represents the PT group, the diagonal bar represents the RT group, the light bar represents before treatment, and the darker bar represents after treatment. ^∗^*P* < 0.05.

**Table 1:** Baseline characteristics of the patients.

	RT (*n* = 27)	PT (*n* = 27)
Age (SD, range)	57.89 (10.08)	52.11 (5.49)
Weeks poststroke (SD, range)	7.00 (2.12)	7.89 (2.57)
Sex (M/F)	18/9	12/15
Side of stroke (L/R)	12/15	18/9
Stroke type (ischemic/hemorrhagic)	15/12	18/9

RT: robot-assisted gait training; PT: physical therapy. Summary of mean (SD) values for demographic variables and clinical measures for the RT and PT groups.

**Table 2:** Changes in Primary and Secondary Outcomes at 2 Weeks.

	PT (*n* = 27) Mean (SD)			RT (*n* = 27) Mean (SD)			Between groups
	Pre	Post	*P*	Pre	Post	*P*	*P*
FMA	17.0 (2.12)	20.22 (2.68)	<0.01	21.3 (5.34)	25.89 (4.60)	0.02	0.26
TUG	26.8 (5.09)	22.43 (3.95)	<0.01	23.4 (6.17)	21.31 (4.92)	0.28	0.97
*Time parameters*							
Stride time	1.75 (0.41)	1.81 (0.42)	0.48	1.84 (0.37)	2.27 (1.19)	0.37	0.90
Single stance	0.60 (0.12)	0.65 (0.17)	0.40	0.66 (0.09)	0.94 (0.69)	0.14	0.63
Double stance	0.33 (0.13)	0.36 (0.13)	0.16	0.37 (0.15)	0.40 (0.33)	0.44	0.15
Swing phase	0.60 (0.12)	0.65 (0.17)	0.40	0.66 (0.09)	0.94 (0.69)	0.14	0.63
Stance phase	1.14 (0.33)	1.16 (0.29)	0.37	1.14 (0.28)	1.39 (0.72)	0.29	0.90
*Space parameters*							
Stride length	122.42 (33.09)	119.49 (30.98)	0.59	102.35 (46.14)	91.74 (39.05)	0.03	0.48
Walk velocity	74.37 (30.10)	71.04 (32.90)	0.31	61.58 (36.55)	54.69 (37.31)	0.03	0.63
Cadence	57.53 (14.33)	55.17 (13.55)	0.44	50.29 (12.00)	53.04 (16.90)	0.44	0.12
Gait width	30.49 (7.97)	33.51 (8.31)	0.02	29.92 (7.02)	33.33 (8.90)	0.21	0.57
Toe out angle	12.86 (5.79)	11.57 (6.50)	0.31	11.53 (9.05)	18.89 (12.02)	0.01	0.00

Summary of mean (SD) values for changes (post, pre) in primary and secondary outcome variables for the RT and PT groups.

## Data Availability

The datasets used in this study are available from the corresponding author on reasonable request.
